# Interleukin-3 prevents neuronal death induced by amyloid peptide

**DOI:** 10.1186/1471-2202-8-82

**Published:** 2007-10-03

**Authors:** Angara Zambrano, Carola Otth, Lorena Mujica, Ilona I Concha, Ricardo B Maccioni

**Affiliations:** 1 Instituto de Bioquímica, Facultad de Ciencias, Universidad Austral de Chile, Chile; 2 Laboratory of Cellular, Molecular Biology and Neuroscience, Millennium Institute for Advanced Studies in Cell Biology and Biotechnology (CBB), Facultad de Ciencias, Universidad de Chile, Chile

## Abstract

**Background:**

Interleukin-3 (IL-3) is an important glycoprotein involved in regulating biological responses such as cell proliferation, survival and differentiation. Its effects are mediated via interaction with cell surface receptors. Several studies have demonstrated the expression of IL-3 in neurons and astrocytes of the hippocampus and cortices in normal mouse brain, suggesting a physiological role of IL-3 in the central nervous system. Although there is evidence indicating that IL-3 is expressed in some neuronal populations, its physiological role in these cells is poorly known.

**Results:**

In this study, we demonstrated the expression of IL-3 receptor in cortical neurons, and analyzed its influence on amyloid β (Aβ)-treated cells. In these cells, IL-3 can activate at least three classical signalling pathways, Jak/STAT, Ras/MAP kinase and the PI 3-kinase. Viability assays indicated that IL-3 might play a neuroprotective role in cells treated with Aβ fibrils. It is of interest to note that our results suggest that cell survival induced by IL-3 required PI 3-kinase and Jak/STAT pathway activation, but not MAP kinase. In addition, IL-3 induced an increase of the anti-apoptotic protein Bcl-2.

**Conclusion:**

Altogether these data strongly suggest that IL-3 neuroprotects neuronal cells against neurodegenerative agents like Aβ.

## Background

The cytokine, Interleukin (IL)-3 is an important regulator which exhibits pleiotropic activities [1]. It is expressed in hematopoietic cells as well in several non-hematopoietic cell types [2-8]. The biological activity of IL-3 is mediated through specific cell surface receptors which are composed of α and β subunits. The α subunit is responsible for the binding of IL-3. The ligand-activated α subunit is associated with the β subunit, which transmits signals across the plasma membrane [9]. IL-3 is known to activate at least three signaling pathways: The Jak/STAT, the Ras/Raf/mitogen-activated protein kinase, and the phosphatidylinositol 3-kinase (PI 3-kinase)/protein kinase B (PKB) pathway. An important PI 3-kinase target is the serine/threonine kinase Akt/PKB, which, mediated by many growth factors [10] (Dudek et al., 1997), is involved in cell survival.

Several studies have demonstrated the presence of IL-3 in the central nervous system [4,5,11]. Although there is evidence indicating that IL-3 is expressed in some neuronal populations [12], its physiological role in these cells is unknown. Some studies [13] demonstrated that IL-3 significantly facilitates sensory neuron survival and stimulates the formation of the neural network *in vitro*, promotes the process extension of cultured cholinergic neurons [14], and that IL-3 exerts a trophic action on hippocampal neurons, rescuing hippocampal CA1 neurons from lethal ischemic damage [15]. However, the mechanism by which IL-3 supports neurons has not yet been determined.

In the nervous system and particularly during development, apoptosis appears to be triggered by trophic factor deprivation. Neuronal apoptosis is likely to occur in Alzheimer's disease (AD), a widespread neurodegenerative disorder that results in progressive dementia [16]. Histopathologically, AD is characterized by the presence of extracellular senile plaques that consist of β-amyloid protein (Aβ) in its fibrillary form, and neurofibrillary tangles [17]. Aβ causes hippocampal and cortical neuronal death *in vitro and in vivo *[18,19]. It has been suggested that Aβ_1–40 _and Aβ_1–42 _downregulate Bcl-2, and that this effect may lead to increased neuronal degeneration during age-dependent stresses [20].

In this study, we provide direct evidence for the functional expression of IL-3 receptors on neurons. We also demonstrated their involvement in the neuroprotective action of IL-3 upon Aβ-neurotoxicity. We demonstrated that receptor activation signals cell survival in the presence of Aβ. Our results suggest that the effect of IL-3 on cortical neurons is mediated by activation of the Ser/Thr kinase Akt and kinase Jak, both important components of anti-apoptotic mechanisms in neurons and other cell types. And worthy of note, IL-3 was able to induce an increase in Bcl-2 protein in these cells.

## Results

### Expression of functional IL-3 receptors in cortical neurons

The expression of both α and β subunits of IL-3 receptor in primary cortical neurons was confirmed using specific antibodies. Immunofluorescence analysis using anti-IL-3rα and anti-IL-3rβ (Fig. 1) antibodies showed clear positive immunostaining in primary cortical neurons. These results suggest that this receptor is expressed in these cells. It is therefore reasonable to assume that these receptors are functional and able to transduce downstream signals. To investigate the possibility that IL-3 treatment produced activation of Jak2, ERK and Akt, lysates from cells treated with IL-3 for various times were subjected to Western blot analysis using anti-phospho-Jak2, -ERK, and -Akt antibodies to detect activated Jak2, ERK and Akt, respectively (Fig. 1B and 1C). Duplicate blots were probed with antibodies recognizing total Jak2, ERK or Akt to verify equal protein loading in the samples. As shown in Fig. 1B, treatment with 5 nM IL-3 led to increased phosphorylation of Jak2 within 10 minutes and this phosphorylation remained elevated for 60 minutes. Treatment with 5 nM IL-3 also weakly activated Akt, an activation which was sustained for 20 minutes. Akt phosphorylation was fast for the first 30 minutes and after 2 h there is an increase that was sustained over 24 h in primary cortical neurons (Fig. 1D).

**Figure 1:** **Expression and activation of IL-3 receptors in cortical neurons**. (A). Primary cortical neurons were incubated with anti-IL-3α subunit (a), anti-IL-3β subunit (b) or without first (c) antibodies followed by incubation with a second antibody conjugated to FITC. Scale bar, 20 μm. (B). Western blot analysis shows Jak2, Akt and ERK phosphorylation in cortical neurons treated with 5 nM IL-3 for the indicated times. (C). Normalized densitometry scans of proteins panel B. (D). Western blot analysis shows Akt phosphorylation in cortical neurons treated with IL-3 for the indicated times. The results are representative of three separate experiments.

Also, ERK activation was evident at 5 minutes and was sustained for over 60 minutes. These results suggest that IL-3 receptors are functional and are able to transduce a signal in response to IL-3.

### Neuroprotective effect of IL-3 on neurons treated with Aβ_1–40_

Several results suggest that aggregated Aβ peptide, as well as the oligomeric forms of this peptide, are highly toxic for a variety of cultured primary neurons and neuronal cell lines. Cortical neurons were treated with different concentrations of the aggregated Aβ peptide (Aβ_1–42_) for 24 h. Aβ was dose-dependently toxic (Fig. 2, panel A), causing up to 40% cell death at 25 μM.

**Figure 2:** **Effect of IL-3 on fibrillary Aβ-induced neurotoxicity in cortical neurons**. MTT, Tripan blue and TUNEL staining analyses were used to determine cell death. (A). Cortical neurons were treated with different concentrations of Aβ peptide for 24 h at 37°C. (B). Neurons were incubated with different concentrations of IL-3 and then treated with 10 μM Aβ. (C). Neurons were incubated with different concentrations of IL-3 in the absence of Aβ. (D). Neurons were incubated with different concentrations of IL-1 and then treated with 10 μM Aβ. Data are mean ± S.E. for three separate experiments performed in duplicate. (E). Cortical neurons were treated with 10 μM Aβ in the absence or presence of 5 nM IL-3 for 24 h at 37°C. TUNEL-positive neurons were visualized by microscopy and the shrunken nuclei are indicating by arrows. (F). Primary cortical neurons were pre-treated with 5 nM IL-3 or 100 μM insulin for 30 min, and then treated with 10 μAβ for 24 h at 37°C. MTT and Tripan blue analyses were used to determine cell death. Data are means ± S.E. for three separate experiments performed in duplicate.

To determine whether IL-3 protects neurons against Aβ, we treated cells with increasing concentrations of IL-3 (0 – 10 nM) 30 min before the assay and maintained a 24 h exposure to aggregated 10 μM Aβ_1–42 _(Fig. 2, panel B). Our results show a dose-dependent reduction in Aβ toxicity following IL-3 treatment, with a clear increase in cell survival at 10 nM IL-3. IL-1 was used as a negative control, having no effect on Aβ toxicity (Fig. 2, panel D). IL-3 alone had no effect on cortical neurons (Fig 2, panel C).

In order to define whether DNA fragmentation occurred in neuronal cultures treated with Aβ in the presence or absence of IL-3, we searched by TUNEL staining. A high number of TUNEL-positive cells with shrunken nuclei and condensed chromatin, as indicated by arrows, were detected in the presence of 10 μM Aβ, whereas the TUNEL- positive cells were far fewer in neuron cells pre-treated with 5 nM IL-3 before 10 μM Aβ treatment (Fig. 2E).

We also proved that the neuroprotective effect on Aβ-neurotoxicity is very similar to that found with insulin treatment (Fig. 2F). This observation suggests that IL-3, similar to insulin may offer trophic support to neurons [21].

### PI3K/Akt participates in IL-3-induced neuroprotection

Activation of Akt requires the phosphorylation of Thr-308 and Ser-473 in the Aktα molecule. In this study, phosphorylation of Ser-473 was used to evaluate the activation of Akt. In order to determine whether Akt activation participates in IL-3-induced neuroprotection we used a specific inhibitor of PI 3-kinase, LY2940002, which is highly selective for PI 3-kinase inhibition. Cortical neurons were pre-treated with 50 μM LY2940002 for 30 min prior to addition of 5 nM IL-3. Cells were then exposed to 10 μM Aβ and incubated for an additional 24 h. These cells were used for Western blot, Tripan blue exclusion and MTT analysis. As shown by Western blot analysis (Figs. 3A and 3B), pre-treatment with LY2940002 blocked the IL-3-evoked Akt activation. Also, LY2940002 blocked the BAD phosphorylation, a downstream effector of Akt, but had no effect on Jak 2 phosphorylation, which is a receptor-associated kinase upstream to Akt. As shown in Fig. 3C, pre-treatment of cells with LY2940002, totally abolished the protective effect of IL-3. The same results were obtained using 100 nM Wortmannin (data not shown). These results suggest that IL-3-induced activation of Akt, by PI 3-kinase, was necessary for protection from Aβ-induced cell death.

**Figure 3:** **Inhibition of PI 3-kinase blocked Akt phosphorylation and IL-3 mediated neuroprotection against Aβ toxicity**. Primary cortical neurons were pre-treated with 50 μM LY2940002 for 30 min before addition of 5 nM IL-3. One hour after addition of growth factor, cells were then exposed to 10 μM Aβ and incubated for an additional 24 h. Cells incubated with vehicle (PBS containing ≤ 0.1% DMSO v/v) and not exposed to IL-3 or Aβ were defined as control cells. Then the cells were used for Western blot and viability analysis. (A) Western blot analysis using phosphorylation-specific antibodies (p-Jak2, p-Akt, and p-BAD), and total anti-Akt1 antibodies. (B). Normalized densitometry scans of proteins (mean ± SEM, *, #, p < 0.05). The student's t-test was used for the statistical analysis of significance of difference. (C). Neuronal death was determined by MTT colorimetric assay and Tripan blue exclusion. Data represent mean ± SEM for three independent experiments (with a minimum of 4–5 wells per group for each experiment).

### Participation of Jak2 in IL-3-induced protection

The members of the family of Jak kinases are associated constitutively with a variety of cytokine receptors, including the IL-3 receptor. Upon binding of the specific ligand to its receptor, Jak kinases are rapidly activated, and their kinase activities are induced to regulate tyrosine phosphorylation of various effectors and to initiate activation of downstream signaling pathways. These pathways include PI3K, MAPK, and NF-κB (nuclear factor-kappa B), leading to cell differentiation, survival and proliferation. To determine whether Jak2 kinase is implicated in IL-3-induced neuroprotection, we used AG490, a highly selective specific inhibitor of Jak2. Cortical neurons were pre-treated for 30 min with 20 μM AG490 before addition of IL-3 and Aβ peptide. AG490 induced a decrease in Jak2 and Akt phosphorylation (Fig. 4A and 4B). Pre-treatment with AG490 totally abolished the protective effect of IL-3 (Fig. 4C). These results suggest that IL-3 induce Jak2 activation, and that this activation is necessary for protection from Aβ-induced death.

**Figure 4:** **Inhibition of Jak2 kinase blocked Akt phosphorylation and neuronal survival by IL-3**. Primary cortical neurons were pre-treated with 20 μM AG490 for 30 min before addition of 5 nM IL-3. One hour after addition of growth factor, cells were exposed to 10 μM Aβ and incubated for an additional 24 h. Cells incubated with vehicle (PBS containing ≤ 0.1% DMSO v/v) and not exposed to IL-3 or Aβ were defined as control cells. Then the cells were used for Western blot and viability analysis. (A) Western blot analysis using phosphorylation-specific antibodies (p-Jak2, and p-Akt), and total anti-Akt1 and anti-Jak2 antibodies. (B). Normalized densitometry scans of proteins (mean ± SEM, *, #, p < 0.05). The student's t-test was used for the statistical analysis of significance of difference. (C). Neuronal death was determined by MTT colorimetric assay and Tripan blue exclusion. Data represent mean ± SEM for three independent experiments (with a minimum of 4–5 wells per group for each experiment).

### Role of ERK in the neuroprotective action of IL-3

Activation of ERK and Akt pathways has been shown to promote cell survival/proliferation after growth factor stimulation and to play a protective role. To investigate ERK involvement, we tested the effect of PD98059 on IL-3-induced neuroprotection. PD98059 is a selective inhibitor of the MEK kinase pathway, kinase upstream of ERK. Cells were pre-treated with 20 μM PD98059 for 30 min prior to addition of IL-3. After addition of IL-3, cells were exposed to 10 μM Aβ and incubated for an additional 24 h. Pre-treatment with PD98059 blocked IL-3-evoked ERK activation, but had no effect on Jak2 and Akt activation (Fig. 5A and 5B). Results are consistent with the notion that Jak2 is a kinase upstream of ERK, and these results therefore suggest that IL-3-evoked Akt activation is not dependent on ERK phosphorylation. Next, we evaluated the ability of IL-3 to promote cell survival in neurons treated with PD98059 for 24 h. As shown in Fig. 5C, PD98059 did not alter the IL-3 effect on Aβ-induced cell death. The results suggest that IL-3 protected against Aβ-induced death by regulating Jak and PI3K/Akt pathways.

**Figure 5:** **Effect of PD98059 on IL-3 mediated neuroprotection against Aβ toxicity**. Primary cortical neurons were pre-treated with 20 μM PD98059 for 30 min before addition of 5 nM IL-3. One hour after addition of interleukin, cells were exposed to 10 μM Aβ and incubated for an additional 24 h. Then the cells were used for Western blot and viability analysis. (A) Immunoblot analysis using phosphorylation-specific antibodies (p-ERK 1/2, p-Jak2, and p-Akt). (B). Normalized densitometry scans of proteins (mean ± SEM, *, #, p < 0.05). The student's t-test was used for the statistical analysis of significance of difference. (C). Neuronal death was determined by MTT colorimetric assay and Tripan blue exclusion. Data represent mean ± SEM for three independent experiments (with a minimum of 4–5 wells per group for each experiment).

### IL-3 induces an increase in Bcl-2 expression

A previous report [20] suggested that Aβ is able to downregulate Bcl-2 protein, a well-established anti-death protein in neurons. Several growth factors, among them IL-3, induce the Bcl-2 expression. To investigate the role of Bcl-2 in the IL-3-induced protection, cells treated with Aβ in the presence or absence of IL-3 were analyzed by Western blot analysis. As shown in Fig. 6, there was a decrease of Bcl-2 protein levels in cells treated with 10 μM Aβ. Cells pre-treated with 5 nM IL-3 1 h before addition of Aβ, presented no decrease in Bcl-2. This suggests that IL-3 is able to maintain Bcl-2 protein levels similar to those in control cells in the presence of Aβ peptide.

**Figure 6:** **IL-3 induces an increase of Bcl-2 protein**. Protein extracts from cortical neurons not exposed to IL-3 or Aβ, were defined as control cells (lane 1), cells treated with 10 μM Aβ in the absence (lane 2) or presence (lane 3) of 5 nM IL-3 and cells treated with IL-3 (lane 4) were analyzed by Western blot using anti-Bcl-2 and anti-actin antibodies. Blots shown are from representative experiments.

## Discussion

It has been proposed that IL-3 has a neuroprotective role, but the mechanism has been poorly described. The data presented here provide strong evidence that IL-3 can act directly on neurons and activate neuronal survival pathways. We demonstrated that IL-3 is a potent inhibitor of neuronal death induced by Aβ_1–42 _exposure. These findings were complemented by kinase phosphorylation studies, including the use of specific inhibitors that identified which survival pathways are activated by IL-3.

Alzheimer's disease (AD) brain is characterized by the selective loss of synapses and neurons. The presence of amyloid plaques composed primarily of aggregated amyloid β-peptide (Aβ), 40 to 42 aminoacids in length, is thought to be the toxic agent in AD [22]. The mechanism by which Aβ induces cell death or apoptosis is not yet clear. Previous authors have suggested that Aβ downregulates survival protein, such as Bcl-2 [20]. Additionally, mutant presinilin 1 (PS1) of familial AD, induces apoptosis, downregulates the survival factor Akt/PKB, and affects several Akt/PKB downstream targets, including glycogen synthase kinase 3 β and β-catenin [23].

However, it has been reported that several factors, such as IGF-I, protect hippocampal neurons from Aβ toxicity. The initial signaling involved in this protection has been shown to involve both ERK and PI 3-kinase-dependent pathways. All these results strongly suggest that Aβ downregulates the natural protective mechanism in neurons, and the activation of some growth factor receptor can protect neurons from Aβ-induced cell death by anti-apoptotic pathways activation.

Previous studies of IL-3 in the central nervous system demonstrated the expression of IL-3 mRNA in neurons of the habenula, hippocampus, cerebral and enthorhinal cortices, and subiculum in normal mouse brain [4], and suggested endogenous IL-3 might be produced by certain neurons [12]. Functional IL-3 receptors are expressed in the central cholinergic neurons and contribute to some physiological roles such as the differentiation and maintenance of these neurons. Also, both hippocampus and cerebral cortex express IL-3rα and β subunits [5].

We demonstrated that primary cortical neurons express IL-3rα and β subunits. Biological response analyses confirmed the presence of functionally active IL-3 receptors, responsive to mouse IL-3 in cortical neurons. Binding of this cytokine to its receptor leads to the stimulation of classical signal transduction pathways, specifically the Jak/STAT pathway, the Ras/MAPK pathway, and the PI 3-kinase/PKB pathway [24]. The data showed that IL-3 induced activation of these pathways in this cell type. In general there was a fast and transient increase of the phosphorylation of p-Jak2 and p-ERK. However, Akt phosphorylation was fast for the first 30 minutes and after 2 h there is an increase that was sustained over 24 h in primary cortical neurons.

The neuroprotective effect of IL-3 against the amyloid was studied by fragmented DNA using TUNEL staining, MTT and Tripan blue exclusion analysis. We demonstrated that IL-3 prevents Aβ-neurotoxicity. IL-3 induces an increase in cell viability of more than 75% in cells treated with Aβ. Our results are consistent with other groups, which have reported that IL-3 has a functional role in some neurons. Some authors have demonstrated that the survival of sensory neurons was significantly supported by IL-3, which also stimulates their morphological differentiation [13]. IL-3 also attenuated neuronal damage caused by free radicals, which are known to be overproduced during and after brain ischemia. Furthermore, IL-3 was able to protect NGF-differentiated neurons from apoptotic cell death caused by NGF withdrawal [25].

We showed that this neuroprotective effect on Aβ-neurotoxicity is similar to that found with insulin treatment. Direct actions of insulin on neurons and neuron-like cells have suggested it may offer trophic or growth factor support to these structures. In some *in vitro *systems, and in some *in vivo *models, a role for direct insulin support for regeneration has been suggested [21].

It has been proposed that IL-3 has a neuroprotective role, but no underlying biological mechanism has been identified. We showed that IL-3 protected against Aβ-induced cell death and activated Akt. A specific inhibitor of PI 3-kinase blocked this activation and abolished protection of Aβ-induced cell death, indicating that activation of Akt was important for IL-3 protection. Activation of Akt protects cells from apoptotic signals such as growth factor withdrawal, cell cycle disruption, and cell detachment [26]. PI 3-kinase has been implicated in the regulation of cell survival in several cell types. In particular, PI 3-kinase is thought to be involved in IL-3-dependent survival, and that a region on the βc receptor important for IL-3-dependent survival is necessary for PI 3-kinase activation. Akt is activated by factors that stimulate PI 3-kinase activity in cells, such as thrombin, platelet-derived growth factor, and insulin [27]. Active Akt can promote cell survival in response to various death stimuli, including withdrawal from growth factors [10]. Here we demonstrated that Akt activity is induced rapidly by the cytokine IL-3 in cortical neurons and that activation of Akt by IL-3 is dependent on the PI 3-kinase activity.

Akt was activated downstream from PI 3-kinase, resulting in the phosphorylation and inactivation of BAD, a principal inducer of cell apoptosis. It has been demonstrated that activated Akt phosphorylates BAD, resulting in its sequestration by cytosolic 14-3-3 proteins [28,29] Because BAD binds to and inhibits the anti-apoptotic actions of Bcl-_XL_, the sequestration of BAD in the cytosol by 14-3-3 proteins results in enhanced survival. This signalling pathway has been shown to play an important role in neuronal development and survival [30].

We also provide evidence that Aβ-induced apoptosis is prevented through the IL-3 induced activation of Jak2. Our findings indicate that IL-3r activation induces Jak2 activation via tyrosine phosphorylation and that this initial event is followed by tyrosine phosphorylation of PI 3-kinase and Akt serine phosphorylation as suggested by the inhibitory effect of AG-490 on the phosphorylation of both proteins. These results are consistent with those reported for hematopoietic cells, in which the kinase domain of Jak2 inhibits cell death and treatment with the Jak2 inhibitor AG-490 reduces phosphorylation of PI 3-kinase, resulting in increased caspase 3 activity and Bax protein in acute myocardial infarction [31]. In addition, activation of neuronal erythropoietin receptors prevents apoptosis by triggering cross-talk between the signaling pathways of Jak2 and the nuclear factor- κB (NF-κB) [31,32].

Activation of ERK and Akt pathways have been shown to promote cell proliferation/survival after growth factor stimulation and to play a protective role. Activation of both ERK and Akt are important steps in cellular responses to a variety of extracellular stimuli [26]. However, we demonstrated that inactivation of the mitogen-activated protein kinase pathway by PD98059, a selective inhibition of mitogen-activated protein kinase/extracellular signal regulated kinase, did not affect IL-3-mediated survival, meaning that the Akt pathway is primarily involved and rendering ERK activation unnecessary for the IL-3-induced survival function. In contrast to our findings, in other cell systems, the inhibition of ERK activation with a dominant-negative MAPKK, suppresses IL-3-dependent survival, in, for example, BaF3 cells [33].

The IL-3-induced targets important for cell survival, seem to be proteins of the anti-apoptotic *bcl-2 *gene family. Expression of *bcl-2 *and *bcl*_*XL *_is rapidly induced by IL-3 or activated Ras in multiple cell types [34,35]. We showed that cells treated with Aβ had decreased Bcl-2 protein levels, consistent with some reports which suggested that Aβ is able to downregulate Bcl-2 protein [20]. However, IL-3 is able to support Bcl-2 protein levels in the presence of Aβ peptide. Overexpression of *bcl-2 *blocks apoptosis induced by IL-3 withdrawal in cell lines [36,37]. Bcl-2 is well established as an anti-death protein in neurons. Bcl-2 can avert survival factor deprivation-induced neuronal apoptosis in sympathetic cervical ganglia, in sensory primary neurons, and in continuous cell lines such as PC12 cells [38].

## Conclusion

In summary, our data constitute the first experimental evidence of the role of IL-3 in neurodegeneration Alzheimer's type. We show that IL-3 prevents neuronal death induced by Aβ peptide and suggest that the specific pathways responsible include activation of PI 3-kinase and Jak2. IL-3 was also able to induce an increase of the anti-apoptotic protein, Bcl-2.

## Methods

### Cell Cultures

Cortical neurons obtained from 16-day-old mice embryos were prepared as previously described [39]. Briefly, embryos were removed from the dams at E16 and placed into Hank's balanced salt solution (1 mM HEPES, pH 7.4, 8 mM NaCl, 0.27 mM KCl, 0.28 mM glucose, 0.02 mM KH_2_PO_4_). Embryonic day 1 was defined as the day of conception established by the presence of a vaginal plug. Embryos were dissected and minced well with scissors. Tissue was dissociated with 0.25% trypsin at 37°C for 15 min and then by mechanical grinding, with a sterile, fire-polished glass Pasteur pipette, in Minimum Essential Media (MEM) supplemented with 10%FBS. The cells were collected by centrifugation and resuspended in a serum-free medium consisting of neurobasal medium (NB) supplemented with B27 and 0.5 mM L-glutamine. Neurons were grown at 37°C in humidified 5% CO2 atmosphere for 7–10 days prior to experimentation. Cortical cells were plated onto coverslips or in 35-mm plastic dishes pre-coated with polylysine (10 μg/ml).

### Preparation of the Aβ fibrils

The Aβ_1–42 _peptide (purchased from Chiron Corporation; Emereville, CA, USA) was subjected to aggregation as described [40]. The Aβ fibrils were concentrated by centrifugation (20.000 × g for 30 min) and resuspended at 1 mg/ml in PBS (137 mM NaCl, 2.7 mM KCl, 10 mM Na_2_HPO_4_, 2 mM KH_2_PO_4_). Aβ concentration was evaluated using the BCA protein assay (Pierce, Rockford, IL. USA) [41].

### Immunofluorescence

Cortical neurons were fixed in 4% paraformaldehyde in PBS for 20 min, washed in several changes of PBS for 10 min, permeabilized in 0.3% Triton X-100 in PBS for 15 min and incubated overnight at 4°C with anti-IL-3rα or anti-IL-3rβ, antibodies (Santa Cruz Biotechnology, Sta. Cruz, CA, USA). After a wash in PBS (three washes, for 15 min each), cells were incubated in fluorescein isothiocyanate-conjugated goat anti-mouse IgG or fluorescein isothiocyanate-conjugated goat anti-rabbit IgG secondary antibodies, for 1 h at room temperature. Fluorescent images were obtained using a Zeiss Axioscope II fluorescence microscope. (Carl Zeiss, Göttingen, Germany).

### Western blot analysis

Cortical neurons were plated at 1 × 10^6 ^cells/cm^2 ^on 35 mm dishes. Cultured cells were exposed to Aβ fibrils and/or interleukins for 24 h, for the described time periods. For the experiments with inhibitors to different kinases, cortical neurons were pre-incubated in the presence or absence of 50 μM LY2940002 (PI3K inhibitor), 100 nM Wortmannin (PI3K inhibitor), 20 μM AG490 (Jak2 inhibitor) or 20 μM PD98059 (MEK inhibitor) for 1 h and then treated for 24 h with Aβ and/or IL-3. Afterwards, cells were homogenized in RIPA buffer (50 mM Tris, pH 7.5, 150 mM NaCl, 5 mM EDTA, 1% NP-40, 0.5% sodium deoxycholate, 0.1% SDS, 100 μg/ml PMSF, 2 μg/ml aprotinin, 2 μM leupeptin, and 1 μg/ml pepstatin) and the protein concentration was determinated by the Bradford analysis [42]. Proteins extracts were resolved by SDS-PAGE (60 μg per lane) in a 10% polyacrylamide gel [43] and transferred to immobilon (Millipore, Bedford, MA, USA). After blocking with 5% non-fat dry milk the membranes were incubated with primary antibodies (Akt, p-Akt, Jak2, p-Jak2, ERK1/2, p-ERK 1/2, Bcl-2, actin, p-BAD antibodies from Santa Cruz Biotechnology, Sta. Cruz, CA, USA) in a 1% BSA in PBS overnight at 4°C. After washing, the membranes were incubated with horseradish peroxidase-conjugated secondary antibodies (Sigma Chemical Co, St. Louis, Mo, USA) for 1 h at room temperature. The antibody blots were developed by chemiluminescence (Amersham, Arlington Heights, IL, USA).

### Viability assays

Primary cortical neurons were seeded in 96-well plates coated with polylysine 10 μg/ml. Then cells were treated with the 10 μM β-amyloid fibrils with or without 5 nM IL-3 or 100 nM insulin, and in the absence or presence of inhibitors 50 μM LY2940002, 100 nM Wortmannin (PI3K inhibitors), 20 μM AG490 (Jak2 inhibitor), and 20 μM PD98059 (MEK inhibitor), as described previously. After 24 h incubation, the mitochondrial activity was measured by the modified 3- [4,5-dimethylthiazol 2-yl]-2,5 diphenyltetrazolium bromide (MTT) assay [44]. This involves determining mitochondrial dehydrogenase activity in intact cells by incubation for 4 h at 37°C with MTT (10 μl de 5 mg/ml MTT solution per well). The reaction was stopped by addition of cell lysis buffer (50% dimethylformamide and 20% SDS, pH 7.4). ΔA values at 550–650 nm were determined the following day, using an automatic microtiter plate reader (Metertech Σ960) and the results were expressed as a percentage of control. The cell viability was also assessed with Trypan blue exclusion.

To measure DNA fragmentation, cells were fixed in freshly prepared 4% paraformaldehyde for 20 min at room temperature and incubated with blocking solution (3% H_2_O_2 _in methanol), then permeabilized in 0.1% Triton X-100, 0.1% sodium citrate on ice for 2 min. Terminal deoxynucleotidyl transferase-mediated dUTP nick-end labeling (TUNEL) was performed using the In situ Cell Death Detection, POD as described by the manufacturer (Roche, Basel, Switzerland).

### Statistical analysis

Data were expressed as the mean ± SEM of the values from the number of experiments performed in triplicate as indicated in the corresponding figures. MTT and Tripan blue data and histograms were evaluated statistically by using the student's t-test, with P < 0.05 considered significant.

## Abbreviations

The abbreviations used are: IL-3, Interleukin 3; Aβ, β-amyloid; JAKs, Janus kinases; STAT, signal transducers and activators of transcription; MAPK, mitogen-activated protein kinase; ERK, extracellular signal-regulated protein kinases; PI 3k, phosphatidylinositol 3-kinase; PKB, protein kinase B; AD, Alzheimer's disease; PBS, phosphate buffered saline; BSA, bovine serum albumin; MTT, 3- [4,5-dimethylthiazol 2-yl]-2,5 diphenyltetrazolium bromide; TUNEL, terminal deoxynucleotidyl transferase-mediated dUTP nick-end labeling.

## Authors' contributions

AZ participated in the study, designing the protocol for the laboratory investigation and coordination of the manuscript. CO participated in the study design and coordination of the manuscript. LM participated in the design of the study. IC and RM conceived the study and participated in its design and helped to draft the manuscript. All authors read and approved the final manuscript.
